# Correlation with Spectral CT Imaging Parameters and Occult Lymph Nodes Metastases in Sufferers with Isolated Lung Adenocarcinoma

This article has been retracted.

**DOI:** 10.1155/2022/5472446

**Published:** 2022-06-25

**Authors:** Ye Liu, Yongkang Nie

**Affiliations:** Department of Radiology, The First Medical Center of PLA General Hospital, Beijing 100058, China

## Abstract

For investigating the correlation with spectral CT imaging parameters and occult lymph nodes metastasis in sufferers with isolated lung adenocarcinoma. The clinic cases data of 352 sufferers with isolated lung adenocarcinoma from January 2019 to January 2022 were assembled. In line with whether the sufferers had occult lymph nodes metastasis, they were taken as a part in the metastasis group (*n* = 172) and the nonmetastasis group. All sufferers were scanned by spectral CT with a dual-phase contrast-enhanced method, and the recording of spectral CT imaging parameters in arteriovenous phase, iodine concentration (IC), water concentration (WC), the slope rate of the spectral HU curve (*λ*HU), the normalized iodine concentration(NIC), the normalized water concentration(NWC), the normalized effective atomic number (Neff-Z)], and receiver operating characteristic (ROC) were employed to analyze the spectral CT imaging parameters of the arteriovenous phase. Evaluation of occult lymph nodes metastases in sufferers with isolated lung adenocarcinoma. The IC, NIC, *λ*HU, and Neff-Z in the arteriovenous phase spectral CT imaging parameters of the metastasis group were obviously smaller than that of the nonmetastasis group, and the discrepancies were statistically obvious (*P* < 0.05). The results of ROC curve analysis manifested that the area under the curve (AUC) of *λ*HU, IC, NIC, and Neff-Z in the CT parameters of the arterial phase were 0. 840 (95%CI : 0. 796–0.883), 0.763 (95% CI : 0.708–0.818), 0.918 (95% CI : 0.888–0.948), 0.778 (95% CI : 0.731–0.826). The AUCs of *λ*HU, IC, NIC, and Neff-Z in the venous phase spectral CT parameters were 0.909 (95% CI : 0.877–0.941), 0.837 (95% CI : 0.792–0.881), and 0.980 (95% CI : 0.968–0.968), respectively. 0.993), 0.792 (95% CI : 0.742∼0.842). Spectral CT imaging parameters have a certain value in evaluating occult lymph nodes metastasis in sufferers with isolated lung adenocarcinoma, which is helpful for doctors to judge the lymph nodes metastasis in sufferers with this disease before surgery.

## 1. Introduction

Lung adenocarcinoma is a type of lung cancer, belonging to nonsmall cell carcinoma and peripheral lung cancer. Lung adenocarcinoma originates from the mucosal epithelium of the smaller bronchi and a few originate from the mucous glands of the large bronchi. There are generally no obvious clinic symptoms in the early stage of the disease and it is often found on chest CT. It is a round or oval mass that generally grows slowly. The occurrence of lymph nodes metastasis is an important evaluation for judging whether the disease has entered an advanced stage. Indicators. The etiology of lung adenocarcinoma is still not completely clear. A large number of medical data show that the risk factors of lung cancer include smoking (including second-hand smoke), asbestos, radon, arsenic, ionizing radiation, halogen alkenes, polycyclic aromatic compounds, and nickel. Adenocarcinoma accounts for approximately 40% of primary lung tumors. It is more likely to occur in women and smokers. If the disease is not controlled in time, the condition deteriorates rapidly, and the tumor occupies most of the lungs, which will have a great impact on the patient's breathing and pose a great threat to the patient's life [1–4]. Isolated lung adenocarcinoma is a special type of lung adenocarcinoma, which only manifests as an isolated pulmonary nodule and is prone to occult lymph nodes metastasis, leading to missed diagnosis and misdiagnosis, delaying the best treatment opportunity, and endangering the patient's life [5, 6]. At present, an X-ray plain film is the main imaging method for screening and diagnosing chest diseases, but this technology is affected by overlapping, and the resolution is relatively poor[7]. Computed tomography (CT) technology has better spatial resolution and density, differential diagnosis and clinical staging in lung cancer, curative effect evaluation of application is becoming more and more widely, but its diagnosis relies mainly on the morphological diagnosis of mediastinal lymph nodes; clinical experience has confirmed the diagnosis way is relatively poor; spectral CT is a more accurate imaging method that has emerged in recent years. It is CT that detects diseases by obtaining more information than conventional CT based on the difference in X-ray absorption of different energies in human tissues. Energy spectrum imaging can obtain different single-energy images of 40∼ 140 keV, which can judge the nature, source, and difference of pathological tissues. Energy spectrum CT can be separated according to the different attenuation of different substances to X-ray, so as to carry out quantitative analysis, can be qualitative of the substances in the area of interest, and can make the radiation dose received by the human body less than ordinary CT, providing more information for early tumor discovery, tumor classification, benign, and malignant tumor identification [8]. By the context on the above research, this study retrospectively analyzed the correlation with spectral CT imaging parameters and occult lymph nodes metastasis in sufferers with isolated lung adenocarcinoma, in order to provide a theoretical basis for more accurate clinic judgment of isolated lung adenocarcinoma.

## 2. Materials and Methods

### 2.1. General Information

352 sufferers with isolated lung adenocarcinoma in our hospital from January 2019 to January 2022 were selected as the research subjects. Sufferers were taken as a part in the metastasis group (*n* = 172) and nonmetastasis group (*n* = 180) in line with whether they had occult lymph nodes metastasis. This research was ratified by the meeting of the atrology Ethics council of hospital, and the imaging tests were obtained with the informed consent of the sufferers and their relations.

#### 2.1.1. Inclusion Criteria

The inclusion criteria were as follows:

1. Sufferers with isolated lung adenocarcinoma diagnosed by pathology and imaging: CT signs were vacuolar sign, bronchial inflatable sign, burr sign, and deep lobulation sign, respectively. Vacuolar sign or bronchial inflatable sign showed coronal low-density shadow in the lesions with different lengths, some with branches, and single isolated round or oval gas density shadow [9].
2. No radiotherapy and chemotherapy before vitality spectral CT examination.

#### 2.1.2. Exclusion Criteria

The exclusion criteria were as follows:

1. Those with contraindications to CT examination
2. Those with other tumors and those allergic to contrast agents
3. Those with unclear CT images and those with incomplete clinic case data

### 2.2. Methods

Examination protocol double-phase (arteriovenous phase) enhanced scan was performed using gemstone spectral imaging (GSI) mode in spectral CT (Discovery CT750 HD, GE Healthcare, USA). We instruct the patient to breathe prior to the examination. The scanning range is from the apex of the lung to the level of the costophrenic angle. Scanning parameter settings are as follows: high and low vitality instantaneous switching voltage (80∼140 keV, time <0.5 ms), current is 360 mA, layer thickness and layer spacing are 5 mm, pitch is 1.375 : 1, rack rotation time is 0.6 s, and the matrix is 512 × 512. Enhanced scan: In line with the patient's body weight, we inject 1.6 ml/kg of non-ionic contrast agent, iohexol injection, into the cubital vein high pressure, and adjust the injection rate in line with the injection volume, and the injection time is ≤ 30 s. For dual-phase scanning, the same layer of thoracic aorta at the level of the main bronchial bifurcation should be selected for monitoring. The trigger threshold is set to 150 HU. After reaching the threshold, the arterial phase image is obtained by delaying scanning for 5.7 s, and the venous phase image is obtained after delaying scanning for 30 s.

Data processing. The original image was reconstructed into a thin-layer image (layer thickness and layer spacing were both 1.25 mm) and then metastasis to the AW4.6 workstation for processing. The analysis software was GSIViewer software, and more than 2 senior attending physicians. Image data were analyzed blindly and dissenting images were accepted after consensus. Selection of lymph nodes region of interest (ROI): calcification, liquefaction, and necrosis should be avoided as much as possible. When the density is uniform, the area of the ROI is greater than 2/3 of the cross-section. If it is not uniform, we select and include all solid components as much as possible.

### 2.3. Observation Indicators

1. Observe and compare the vitality spectral CT imaging parameters in the arteriovenous phase (arteriovenous phase iodine concentration(IC), water concentration(WC), the slope rate of the spectral HU curve (*λ*HU), normalized iodine concentration (NIC), normalized water concentration (NWC), normalized effective atomic number (Neff-Z)), calculation formula: *λ*HU = (40 keV single-energy CT value-100 keV single-energy CT value)/60; NIC = ROI iodine concentration of lymph nodes/Iodine concentration in thoracic aorta ROI; NWC = water concentration in lymph nodes ROI/water concentration in thoracic aorta ROI; Neff-Z = valid nuclear figure of lymph nodes/valid nuclear figure of descending aorta
2. To analyze the value of spectral CT imaging parameters in arteriovenous phase in evaluating occult lymph nodes metastasis in sufferers with isolated lung adenocarcinoma

### 2.4. Statistical Methods

SPSS 22.0 AutoCAD was employed for info analysis. Measurement data were expressed by means of (mean ± SD), and *t*-test was employed for comparison. Receiver operating characteristic(ROC) analysis of spectral CT imaging parameters in the arteriovenous phase for the evaluation of occult lymph nodes metastasis in sufferers with isolated lung adenocarcinoma. The area under the curve (AUC) and the 95% confidence interval were calculated, and the cutoff point value was taken as the corresponding value of the cutoff point corresponding to the maximum Youden index (sensitivity + specificity-1). Discrepancies were considered statistically obvious at *P* < 0.05.

## 3. Results

### 3.1. Contrast by Two Groups of Arterial Phase Spectral CT Parameters

There was no obvious discrepancy in WC and NWC in the arterial phase Spectral CT parameters with the metastasis group and the nonmetastasis group (*P* > 0.05). The *λ*HU, IC, NIC, and Neff-Z values in the arterial phase spectral CT parameters of the metastasis group were obviously smaller than those of the nonmetastasis group, and the discrepancies were statistically obvious (*P* < 0.05), as shown in Table 1.

### 3.2. Contrast by Venous Phase Spectral CT Parameters with the Two Groups

There was no obvious discrepancy in WC and NWC in the venous phase vitality spectral CT parameters with the metastasis group and the nonmetastasis group (*P* > 0.05), which were obviously smaller than those in the nonmetastasis group, and the discrepancies were statistically obvious (*P* < 0.05), as shown in Table 2.

### 3.3. ROC Curve Analysis of Arterial Phase Spectral CT Parameters in Evaluating Occult Lymph Nodes Metastasis in Sufferers with Isolated Lung Adenocarcinoma

The results of ROC curve analysis manifested that the AUCs of *λ*HU, IC, NIC, and Neff-Z in the CT parameters of the arterial phase were 0.840 (95% CI : 0.796–0. 883), 0.763 (95% CI : 0.708–0.818), 0.918 (95% CI : 0.888–0.948), and 0.778 (95% CI : 0.731–0.826), as shown in Table 3 and Figure 1.

### 3.4. ROC Curve Analysis of Venous Phase Spectral CT Parameters in Evaluating Occult Lymph Nodes Metastasis in Sufferers with Isolated Lung Adenocarcinoma

The ROC curve analysis results manifested that the AUCs of *λ*HU, IC, NIC, and Neff-Z in the venous phase vitality spectral CT parameters were 0.909 (95% CI : 0.877–0.941), 0.837 (95% CI : 0.792–0.881), 0.980 (95% CI : 0.968∼0.993), and 0.792 (95% CI : 0.742∼0.842), as shown in Table 4 and Figure 2.

### 3.5. CT Images of Typical Cases

The CT image of a 67 year-old male with lung adenocarcinoma around the apical segment of the right upper lobe with mediastinal lymph node metastasis is shown in Figure 3.

## 4. Discussion

Lung cancer is one of the most common malignant tumors in the world and ranks among the top causes of death from malignant tumors in urban populations in the world. Its pathological types mainly include squamous cell carcinoma, adenocarcinoma, and neuroendocrine tumor. In 40–55% of all lung cancers, the early symptoms are mostly occult, and the late symptoms are complex and diverse, lacking specificity, and the early surgical treatment effect is better. Losing the opportunity for surgery, the 5 year survival rate is extremely low, and it is a serious threat to the patient's life [10, 11]. Isolated lung adenocarcinoma belongs to one of the types of lung adenocarcinoma, and judging whether lymph nodes metastasis is of great significance to clarify the patient's condition and improve clinic prognosis. Conventional CT examination has become the preferred imaging method for the diagnosis and differential diagnosis of lung cancer at this stage, but it mainly relies on the morphological changes of the lesions for diagnosis, resulting in high false-negative and false-positive rates in the diagnosis of lymph nodes metastasis. Spectral CT imaging technology is an excellent crystallization of the continuous optimization and development of imaging technology, which can improve more imaging information than conventional CT [12–14]. This study attempted to investigate the correlation with spectral CT imaging parameters and occult lymph nodes metastasis in sufferers with isolated lung adenocarcinoma, and the report is as follows.

The results of this study manifested that IC, NIC, *λ*HU, and Neff-Z values in the arteriovenous phase spectral CT imaging parameters of the metastasis group were obviously smaller than that of the nonmetastasis group, and the discrepancies were statistically obvious. The spectral CT imaging parameters with obvious discrepancies were analyzed by the ROC curve, and the results manifested that *λ*HU, IC, NIC, and Neff-Z values in the spectral CT parameters in the arteriovenous phase all had better effects on the occult lymph nodes metastasis in sufferers with isolated lung adenocarcinoma. Assessed value. To explore the reason, spectral CT imaging technology replaces conventional CT detectors with artificial gem material detectors, which can realize conversion in a short time. Then, the preliminary analysis is completed by the X-ray absorption coefficient of the base material, and then the material is separated to obtain the material content in the tissue and obtain the extent attenuation curve. By analyzing the correlation with the absorption coefficient and change of different tissues, the A qualitative diagnosis was made [15–18]. Compared with conventional CT, spectral CT adds functional analysis, which can identify small lesions and small nodules that cannot be identified by conventional CT, and provide more abundant and comprehensive imaging information for clinic diagnosis. Studies have shown that a large quantity of microvascular dilations appear in metastasis lymph nodes, but they belong to dysplasia, with more damaged vessel walls and narrow lumen; nonmetastasis lymph nodes are stimulated by regulatory factors, and there will also be obvious vascular proliferation, But its vascular tissue structure is complete [19–22]. Moreover, the internal structure of metastasis lymph nodes is abnormal due to tumor cells, and a large quantity of tumor cells destroy the structure of their small blood vessels, resulting in reduced blood supply [23–25]. Water widely exists in various tissues and organs and iodine contrast agents are mainly distributed in diseased blood vessels. By using iodine-water as the base substance in this study, the vascular structure and blood supply of various organs and tissues can be fully reflected, and the presence of metastasis lymph nodes can be identified.

This study is a regression study, which has certain limitations and may have retrospective bias. The cutoff value of the ROC curve analysis has not been demonstrated in practice, and the sample size of this study is small. Accurate conclusions still need to be confirmed by further multicenter, large-sample prospective studies.

## 5. Conclusions

Spectral CT imaging parameters have a certain value in evaluating occult lymph nodes metastasis in sufferers with isolated lung adenocarcinoma, which is helpful for doctors to judge the lymph nodes metastasis in sufferers with this disease before surgery, In the future, it is expected to be combined with other examination methods to further improve the diagnosis of isolated lung adenocarcinoma.

## Figures and Tables

**Figure 1:** ROC curve of arterial phase spectral CT parameters in evaluating occult lymph nodes metastasis in sufferers with isolated lung adenocarcinoma.

**Figure 2:** ROC curve of venous phase spectral CT parameters in evaluating occult lymph nodes metastasis in sufferers with isolated lung adenocarcinoma.

**Figure 3:** CT image of patient. (a) Pulmonary window; (b) mediastinal window; (c, d) arterial phase and venous phase: nodules in the apical segment of the right upper lobe, about 19 ∗ 16 mm in size, with lobulated edges and burrs, relatively uniform density, CT value of about 13–30 HU, visible blood vessels Cluster sign and pleural depression sign, bronchiectasis is seen around, the enhancement scan is unevenly enhanced, the solid part is obviously enhanced, and the CT value is about 43–60H; (e, f)lymph nodes, moderately enhanced on contrast-enhanced scan (arrows).

**Table 1:** Contrast by spectral CT parameters of arterial phase with two groups (mean ± SD).

Argument	Metastasis group (*n* = 1 72)	Nonmetastasis group (*n* = 180)	*t*	*P*
*λ*HU	1.81 ± 0.12	2.06 ± 0.21	13.630	<0.001
IC	18.80 ± 0.80	20.38 ± 2.55	7.769	<0.001
WC	1030.85 ± 14.60	1032.54 ± 13.78	1.117	0.265
NIC	0.21 ± 0.01	0.24 ± 0.02	17.673	<0.001
NWC	1.02 ± 0.02	1.03 ± 0.07	1.804	0.072
Neff-Z	8.63 ± 0.08	8.73 ± 0.10	10.331	<0.001

**Table 2:** Contrast by venous phase spectral CT parameters with two groups (mean ± SD).

Argument	Metastasis group (*n* = 1 72)	Nonmetastasis group (*n* = 180)	*T*	*P*
*λ*HU	2.34 ± 0.05	2.48 ± 0.10	16.495	<0.001
IC	20.04 ± 1.06	22.33 ± 2.03	13.177	<0.001
WC	1027.47 ± 11.50	1025.62 ± 16.21	1.230	0.220
NIC	0.42 ± 0.01	0.46 ± 0.02	23.565	<0.001
NWC	1.01 ± 0.04	1.02 ± 0.06	1.831	0.068
Neff-Z	8.63 ± 0.04	8.72 ± 0.11	10.111	<0.001

**Table 3:** ROC curve analysis of arterial phase spectral CT parameters in evaluating occult lymph nodes metastasis in sufferers with isolated lung adenocarcinoma.

Argument	AUC	*P*	95% CI	Critical value	Sensitivity (%)	Specificity (%)
*λ*HU	0.840 _	<0.001	0.796 ∼ 0.883	1.88	80.50	74.20
IC	0.763 _	<0.001	0.708 ∼ 0.818	20.28	54.90	72.40
NIC	0.918	<0.001	0.888 ∼ 0.948	0.21	90.20	78.80
Neff-Z	0.778	<0.001	0.731∼0.826	8.66	72.00	66.70

**Table 4:** ROC curve analysis of venous phase spectral CT parameters in evaluating occult lymph nodes metastasis in sufferers with isolated lung adenocarcinoma.

Argument	AUC	*P*	95% CI	Critical value	Sensitivity (%)	Specificity (%)
*λ*HU	0.909	<0.001	0.877∼0.941	2.42	61.00	90.90
IC	0.837	<0.001	0.792∼0.881	21.16	67.10	93.90
NIC	0.980	<0.001	0.968∼0.993	0.42	93.90	71.20
Neff-Z	0.792	<0.001	0.742∼0.842	8.68	56.10	86.40

## Data Availability

The simulation experiment data used to support the findings of this study are available from the corresponding author upon request.
